# Green and Energy-Saving Ecological Reconstruction Design of Existing Buildings in Cities in Severe Cold Areas

**DOI:** 10.1155/2022/3125425

**Published:** 2022-09-28

**Authors:** Huan Zhang, Tao Yang

**Affiliations:** ^1^Department of Civil Engineering, School of Engineering, Zhengzhou Technology and Business University, Zhengzhou, Henan Province 451400, China; ^2^Henan University of Animal Husbandry and Economy, School of Energy and Intelligence Engineering, Zhengzhou, Henan Province 450000, China

## Abstract

In order to improve the overall structural stability and thermal insulation capacity of existing buildings in severe cold areas, green energy-saving ecological transformation methods of existing buildings in severe cold areas are proposed. The concrete stress analysis method of the joints in the frame is used to calculate the bearing capacity and prestress of the beam-column joints. Based on the method of parameter analysis, the calculation model of shear capacity is established. The embedded anchoring method is adopted to realize the equal strength connection of beam-column joints. Increase the unbalanced moment between reinforcement and steel plate, and improve the stability and reliability of beam-column joint fixation. The overall structural optimization method of joint shear performance is adopted to reduce the distance between lap reinforcement and steel plate, so as to realize the green energy-saving ecological transformation design of existing urban buildings in severe cold areas. The test results show that the service stress and tensile resistance of the reconstructed existing building area are higher than 60, the tensile capacity is good, and the slip of the lap reinforcement is effectively controlled. At the same time, this method improves the stability of beam-column elements and the overall thermal insulation performance of existing buildings in cities in severe cold areas. The next research will focus on the transformation of other structures.

## 1. Introduction

In recent years, with China's great emphasis on the ecological environment, the concepts of low-carbon cities and green energy-saving buildings have been gradually popularized. With the constant improvement of China's green energy-saving construction, the growth of building energy consumption has been effectively restrained. However, there are still some problems, such as people's ignorance of building energy-saving ideas, imperfect building energy-saving renovation methods and technologies, lack of energy-saving ideas in building construction [1, 2], and inadequate supervision and management of energy-saving renovation.

At present, for residential units, there are often some problems, such as unreasonable layout of residential buildings, inefficient use of space, ventilation and lighting of residential buildings failing to meet the requirements of residents, wasting a lot of energy and so on. Therefore, the application of low-carbon concept and low-carbon technical measures in planning and architectural design to build energy-saving green communities and energy-saving buildings is not only of great significance to China's energy conservation and utilization [3–6], but also significantly improves the living environment of residents. By optimizing the fixed design of beam-column joints of existing buildings in cities in severe cold areas, the overall stability and stress reliability of the building structure are improved, and it is of great significance to study the green energy-saving ecological transformation method of existing buildings in cities in severe cold areas, which is of great concern to people.

China's research on the application of low-carbon energy-saving theory and space syntax in building energy-saving renovation is still insufficient, and the current research results in this area are also lacking, and have not formed a complete system. This study systematically sorts out the application theory of low-carbon energy conservation and the practice method of spatial syntax by analyzing the Reference, reports and excellent cases of the implementation and application of low-carbon energy conservation concepts at home and abroad, perfecting and enriching the energy conservation theory of existing residential areas and residential buildings, and supporting the construction of low-carbon energy-saving communities in China. In this study, the spatial syntax theory is applied to the quantitative and visual analysis of existing residential areas, which can more intuitively analyze the energy-saving transformation of residential areas and buildings. The comprehensive application of space syntax and low-carbon energy-saving theory will provide a new direction and path for the renovation of low-carbon energy-saving residential areas in the future. The design of green energy-saving ecological transformation of existing buildings in cold regions is based on the optimization design of mechanical parameters of beam-column joints of existing buildings in cold regions, and the optimization of green energy-saving ecological transformation of existing buildings in cold regions is realized by combining numerical simulation and mechanical analysis. At present, for the green and energy-saving ecological transformation methods of existing buildings in cities in severe cold areas, the anchor joint fixing method, the foundation pit fixing method, and the tensile steel bar strain stability fixing method are mainly adopted, and the double steel plate concrete composite wall design method is adopted to realize the stability control of beam-column joints of existing buildings in cities in severe cold areas.

Reference [7] proposed a three-dimensional virtual technology for energy-saving space design of green buildings. Use the three-dimensional virtual model of green building and Geographic Information System (GIS) technology to obtain the relevant information of green energy-saving building. It is imported into DeST-c software to simulate the heat balance of green buildings. Reference [8] by analyzing the advantages of BIM Technology and applying it to green buildings, simulates and analyzes the important evaluation parts of green buildings, such as indoor lighting, outdoor acoustic environment simulation, indoor acoustics and outdoor wind environment simulation, and optimizes them in time, so as to achieve the purpose of energy-saving and eco-friendly design of green buildings. Reference [9] discusses the theoretical research trends of Engineering Procurement Construction (EPC) mode, risk sharing, incentive mechanism and energy efficiency labeling system of energy-saving transformation of existing buildings abroad from the perspective of market operation of energy-saving transformation of existing buildings. This paper summarizes the practical characteristics of the operation of the foreign existing building energy-saving reconstruction market from four aspects: laws and regulations, information transmission mechanism, incentive policies, and financing environment. This paper combs the theoretical research results of the operation of China's existing building energy-saving reconstruction market from four aspects: government supervision, behavior strategy, income distribution and financing mode, and summarizes the practical work of the operation of China's existing building energy-saving reconstruction market. Based on the perspective of market governance, starting with the analysis of the particularity of the market governance of the green transformation of existing buildings, this paper demonstrates the theoretical value and practical urgency of the research on the optimization and operation of the market governance system of the green transformation of existing buildings. However, the overlapping intensity of this method in the green, energy-saving, and ecological transformation of existing buildings in cities in severe cold areas is not high. Reference [10] aimed at the typical residential space plane type of existing residential areas in the north, taking Taishan community in Dalian City, Liaoning Province as the research object, the grass hopper platform was used to conduct quantitative simulation analysis and Research on the impact of the target residential building shape, surrounding building types, building spacing and orientation parameters on the operating energy consumption and carbon reduction of existing residential areas. By analyzing 240 simulation cases constructed by parameter transformation, the operating energy consumption of typical residential types under the current envelope conditions under the real layout of existing residential areas in the north is obtained. According to the 50% energy-saving requirements in jgj26-2018 “design standard for energy efficiency of residential buildings in severe cold and cold regions,” a series of passive energy-saving transformation means of external wall insulation and replacement of doors and windows for buildings in existing residential areas are simulated parametrically to quantitatively evaluate the energy-saving and carbon reduction effects after transformation. But this method costs a lot of money.

The vast majority of existing buildings belong to non-energy-saving high-energy buildings. In the energy-saving transformation of existing buildings, local practices basically focus on large-scale public buildings and government office buildings with high-energy consumption, as a breakthrough in energy-saving transformation. Therefore, this paper proposes a green and energy-saving ecological transformation method of existing buildings in cities in severe cold regions based on the overall structural optimization of node shear performance. Firstly, in assembling the integral shear wall structure, the concrete stress analysis method of the joints in the frame is adopted, the embedded anchorage method is adopted, and the prestressed reinforcement degree analysis and yield response analysis are combined to realize the equal strength connection of the beam-column joints of the existing urban buildings in severe cold areas. Then, the static monotonic tensile test method is adopted to increase the moment of force between steel bars and steel plates, improve the stability and reliability of the beam-column joints, and the overall structural optimization method of the shear performance of the joints is adopted to reduce the distance between the overlapping steel bars and steel plates. Finally, the experimental test shows the superior performance of this method in improving the green energy-saving ecological transformation ability of existing urban buildings in severe cold areas.

## 2. Theory of Parameter Analysis Method

Parameter analysis method is widely used in various reservoir parameters. Through cluster analysis and discriminant analysis, the types of flow units in the study area are reasonably divided, and the discriminant functions of various flow units are established to identify the unit types. These parameters mainly include porosity, permeability, median grain size, shale content, formation coefficient, net-gross ratio, saturation, conductivity coefficient, storage coefficient, pore throat radius, pore throat ratio, and cross-well flow capacity index.

### 2.1. IFCI Method of Inter-Well Fluidity Index

Cans identifies the flow unit by using the cross-well flow capacity index Interwell Flow Capacity Index (IFCI). IFCI is defined as the ratio of flow between two adjacent wells. The denominator is the flow rate of high permeability layer. The results show that if the two wells are located in the same flow unit, the ratio of formation coefficient of the two wells has a good correlation with its flow rate ratio. Otherwise, the correlation is poor. Therefore, the distribution range and connectivity of flow units can be judged.

### 2.2. Repeat the Formation Test Repeat Formation Tester (RFT) and Tracer Test Method

Identification of flow unit by repeated formation test and tracer test. The main principle is to identify the flow unit according to the measured pressure change and tracer concentration change.

### 2.3. Production Pressure Difference Method

Prediction of flow unit by production pressure difference. According to the flow of fluid in oil–water two-phase obeying Darcy's law, the calculation formula of production pressure difference of flow unit is established. This method can avoid the contradiction between resource waste caused by shut-in pressure measurement and less pressure measurement data by layers, and its accuracy depends on the accuracy of parameter selection and the reliability of flow unit division.

### 2.4. FIS Method of Inclusion Stratigraphy

Fluid Inclusion Stratigraphy (FIS) is used to identify oil–water interface and seepage barrier, and production logging and pressure data are used to identify flow units. It is worth noting that when the physical and chemical properties of fluid inclusions between adjacent wells are different, it can indicate the existence of barrier layer. However, when there is no difference in physical and chemical properties of fluid inclusions between adjacent wells, it cannot be concluded that the barrier layer does not exist.

## 3. Quantitative Analysis of Green Energy-Saving Transformation of Existing Urban Buildings in Severe Cold Areas

### 3.1. Existing Buildings in Cities in Severe Cold Areas

Based on the research and analysis of domestic and foreign cases, it is concluded that domestic green low-carbon energy-saving residential communities usually pay attention to the application of low-carbon energy-saving concept from the early planning and design stage. In the construction stage, domestic residential areas also adopt construction methods such as assembly to reduce energy consumption and waste of resources in the construction stage. Many technologies and methods are also used in the residential operation stage, which play a substantial role in the energy conservation and utilization of the whole residential area, but the public participation is not high and the enthusiasm is not strong. Compared with foreign low-carbon energy-saving communities, they have invested a lot of financial resources and manpower in the active energy-saving and passive energy-saving design of residential areas, and paid great attention to public participation and the cultivation of residents' low-carbon energy-saving concept in the whole process, which is very worthy of our reference [11–14]. Combined with the stress parameter analysis method of beam-column joints of existing buildings in cold regions, the connection model of concrete foundation and double steel plate composite wall joints of existing buildings in cold regions is established. Firstly, among the three most basic syntactic models, such as convex spatial model, visibility model, and linear element model, the most appropriate spatial syntactic model is selected according to different scales. In the scale range of residential area, the linear factor model is selected for analysis. In this study, the line segment model of linear elements is used for analysis, the axis map representing the street is drawn according to the syntax theory, and the spatial network indicators, such as traversal degree, integration degree, and understandability are analyzed through operation. In the spatial syntax Depthmap software, each line segment (each spatial element) will have a series of spatial network indicator data after calculation. According to the size of these data values, Arrange with color gradient, visualize it in a more intuitive way, compare and analyze it, and get the process diagram of axis model verification, as shown in Figure 1.

Verify through the node count in the software. If the value of node count is positive, it indicates that the drawing is correct, and the color of the line segment is green. If the value is negative, the model is wrong and the color of the line segment is red.

Using reinforced concrete raft as foundation, combining embedded anchoring and embedded anchoring methods, the anchoring connection module of beam-column joints of existing buildings in cities in severe cold areas is established. According to three anchoring forms, double steel plate concrete composite wall configuration method is adopted, and bolts on both sides of beam-column joints of existing buildings in cities in severe cold areas are used to achieve anchoring. Considering raft foundation, embedded steel plates of beam-column joints of existing buildings in cities in severe cold areas are perforated. The cracks of reinforced lap specimens are fixed by anchor bolts, and the ribbed steel bars are lapped in concrete by embedded anchorage. Through strain detection and mechanical parameter analysis of tensile steel bars and steel plates, the wall-reinforced concrete foundation parameters of beam-column joints of existing buildings in cities in severe cold areas are determined. Based on the code for design of building thermal insulation (GB 50011-2010), the thermal insulation design of beam-column units of existing buildings in cities in severe cold regions is carried out. In AISC N690-12, the tensile reinforcement is configured in combination with the technical standard requirements of cylindrical head welding nails for arc stud welding (GB/T 10433-2002).

### 3.2. Constitutive Relationship of Beam-Column Joint Materials of Existing Buildings in Severe Cold Areas

Through field investigation, case comparison and spatial syntax model analysis, this paper analyzes the constitutive relationship of beam-column joints of existing buildings in severe cold regions.

In order to comprehensively consider the green energy-saving design level of buildings in residential areas and the maintenance degree of green environment in residential areas, the building materials of residential buildings and the property management of residential areas are also analyzed. In the assembled integral shear wall structure of existing buildings in cities in severe cold areas, the concrete stress analysis method of the joints in the frame is adopted, and the spatial structure, planning layout and traffic flow lines of two existing residential areas are analyzed at the macro level. For the overall layout and traffic, through the axis model of two existing residential areas, it is analyzed according to two indicators: selectivity and integration. According to the axis model established by the urban road network, the roads represented by each axis have corresponding index values. The values are arranged according to the size, and the color is attached for visual analysis. In the model, the red, yellow and blue axes represent high, medium, and low index values in turn. Among them, the main syntactic index of axis: Choice〉 indicates the potential of axis to attract crossing traffic. Integration represents the traffic accessibility of the axis. In assembling the integral shear wall structure, the concrete stress analysis method of the joints in the frame is adopted to calculate the bearing capacity and prestress of the beam-column joints of the existing buildings in cities in severe cold areas, and the constitutive model of the materials of the beam-column joints of the existing buildings in cities in severe cold areas is constructed [15–17]. The embedded anchorage method is adopted, combined with the analysis of prestressing tendons and yield response, to realize the equal strength connection of the beam-column joints of the existing buildings in cities in severe cold areas. The bending stress model is as follows:

(1) $$\begin{array}{c} f_{t}=\frac{\Delta V_{t}}{V_{t1}}=\frac{V_{t1}-V_{u1}}{V_{t1}}. \end{array}$$

In the above formula, *V*_*t*1_ represents the internal force of tensile reinforcement configuration of existing buildings in cold regions relative to the node performance, *V*_*u*1_ represents the standard anchorage length of reinforcement, and Δ*V*_*t*_ represents the distance between lap reinforcement and steel plate of existing buildings in cold regions. The static loading test method is adopted to analyze the correction factor of lap reinforcement diameter as follows [18]:

(2) $$\begin{array}{c} d_{i}=d_{ei}+d_{pti}, \end{array}$$

where in *d*_*ei*_ is the hysteretic coefficient of the cross-section and steel plate of the existing building specimen in the cold area city, and *d*_*pti*_ represents the buckling relation of large local deformation. The template parameters on both sides of the existing building concrete pouring in the cold area city, and the stress parameters of the anchoring reinforcement are:

(3) $$\begin{array}{c} \left\{\begin{array}{c} b_{20}\left(t;\lambda \right)=\frac{1}{2}\left(1-\lambda t\right){\left(1-t\right)}^{3},\\ b_{21}\left(t;\lambda \right)=\frac{1}{2}\left[1+\left(\lambda +3\right)t-3\left(\lambda +1\right)t^{2}+4\lambda t^{3}-2\lambda t^{4}\right],\\ b_{22}\left(t;\lambda \right)=\frac{1}{2}\left(1-\lambda +\lambda t\right)t^{3}, \end{array}\right. \end{array}$$

where in *λ* is the index of compression and tensile damage of existing buildings in cities in severe cold areas, and *t* is the volume stirrup ratio of energy-saving ecological renovation of existing buildings in cities in severe cold areas. Considering the size and loading capacity of the loading device, it is found that the index coefficient of tensile damage of beam-column joints of existing buildings in cities in severe cold areas satisfies *u* : *I* × *IR*^*d*^⟶*IR*, and the elastic modulus of concrete of existing buildings in cities in severe cold areas is:

(4) $$\begin{array}{c} k_{z}^{g}\left(t,\tau \right)=k_{z}\left(t,\tau \right)=z\left(t+\frac{\tau }{2}\right)z^{*}\left(t-\frac{\tau }{2}\right), \end{array}$$

where in *s* ≥ 0, 1/*p*=1/*p*_1_+1/*p*_2_=1/*p*_3_+1/*p*_4_. The index coefficients of compressive and tensile damage of existing building concrete in cities in severe cold areas are analyzed. When ∃*x*_0_ ∈ *R*_2_, the tensile damage index of concrete in steel tube:

(5) $$\begin{array}{c} i=\underset{j}{\max}\left\{\frac{P\left(Y|\lambda_{j}\right)}{P\left(Y|\lambda_{j}\right)>P\left(Y|\lambda_{T}\right)}\right\}, \end{array}$$

where in *P*(*Y|λ*_*j*_) is the biaxial compressive yield strength of existing urban buildings in severe cold areas, *P*(*Y|λ*_*j*_) is the uniaxial tensile stress of existing urban buildings in severe cold areas, and *P*(*Y|λ*_*T*_) is the initial elastic modulus. If *a* > 1, the constitutive relation model of beam-column joints of existing urban buildings in severe cold areas is established, and the constitutive relation analysis of beam-column joints of existing urban buildings in severe cold areas is realized under uniaxial stress.

## 4. Optimization of Green Energy-Saving Ecological Transformation of Existing Buildings in Cities in Severe Cold Areas

### 4.1. Analysis of Overall Structural Parameters of Shear Performance of Joints

On the basis of the above-mentioned constitutive relation model of beam-column joints of existing buildings in cities in severe cold areas, the overlapping force transmission analysis of beam-column joints of existing buildings in cities in severe cold areas is carried out by adopting the arrangement of overlapping steel bars, and the stress parameter analysis model of beam-column joints of existing buildings in cities in severe cold areas is established by analyzing the bearing capacity, stiffness, and other parameter information of beam-column joints of existing buildings in cities in severe cold areas. Steel plates are welded at the bottom of steel plates, Calculate the stress parameters of the anchorage zone between column and foundation, build the calculation model of shear bearing capacity, adopt the embedded anchorage method, and combine the analysis of prestressing tendons and yield response to obtain the longitudinal strength of the beam-column joints of existing urban buildings in severe cold areas, and establish the finite element model of the beam joints [19]. The compressive stress of existing urban building concrete in severe cold areas is as follows:

(6) $$\begin{array}{c} \varphi \left(a,t,s,b\right)=\sum_{x=\left(p/2\right)}^{\left(p/2\right)-1}\varphi_{x}\left(a,t,b\right)v^{-wx\beta },\\ x=-\frac{P}{2},\cdots ,\frac{P}{2}-1, \end{array}$$

where in *P* is the applied prestress, *φ*_*x*_ is the anchor parameter of the existing buildings in the cold region, *v* is the prestress, *b* is the structural fitting parameter, *a* is the yield response of ecological design, and *t* is the constitutive model parameter.

The calculation model of shear capacity includes the main influencing factors, such as beam geometric size, shear span ratio, stirrup ratio, axial prestress, concrete strength, load form, and so on. During the construction, 987 beams without web reinforcement were selected, including 531 beams with web reinforcement, 136 beams without web reinforcement, and 42 beams with web reinforcement under uniform load. Other prestress, bearing capacity, concrete strength, load, and other parameters are set in the test.

Therefore, combined with the finite element analysis of composite frame joints, the relationship between compressive stress and compressive strain is shown in Figure 2.

According to the relationship between compressive stress and compressive strain of green energy-saving ecological renovation of existing buildings in cities in severe cold areas shown in Figure 2, the finite element simulation method is adopted to test the lap joint force transmission between steel plates and steel bars. The solution domain is considered to be composed of many small interconnected subdomains called finite elements, and a suitable approximate solution is assumed for each element, so that the compressive stress satisfying conditions of green energy-saving ecological renovation of existing urban buildings in severe cold areas can be deduced and solved, and then the stress situation of tensile steel bars can be obtained. In the finite element analysis model of composite frame joints, the relationship between compressive stress and strain of roots is distributed, and the anchorage method of existing buildings in cities in severe cold areas is adopted to weld both ends of tensile steel bars on steel plates. The stress of tensile steel bars in different positions on green energy-saving ecological renovation of existing buildings in cities in severe cold areas is analyzed, and the results are as follows:

(7) $$\begin{array}{c} \left\{\begin{array}{c} x_{i}^{\left(k+1\right)}=\frac{1}{a_{ii}}\left(b_{i}-\sum_{j=1}^{i-1}a_{ij}x_{j}^{\left(k+1\right)}-\sum_{j=i+1}^{n}a_{ij}x_{j}^{\left(k\right)}\right),\\ a_{ij}\neq 0,i=1,2,\cdot \cdot \cdot ,n, \end{array}\right. \end{array}$$

where in *a*_*ii*_ is the stress–strain joint distribution characteristic of green energy-saving ecological transformation of existing buildings in cold regions, *b*_*i*_ is the deviation value of green energy-saving flow potential of existing buildings in cold regions, *x*_*j*_^(*k*)^ is the expansion angle of concrete, and *x*_*j*_^(*k*+1)^ is the strain corresponding to uniaxial compression of green energy-saving ecological transformation of existing buildings in cold regions. According to the analysis of the overall structural parameters of shear performance of beam-column joints of existing buildings in cold regions, the standard anchorage length of steel bars is calculated by the method, and the influence of anchorage length on the performance of beam-column joints of existing buildings in cold regions is analyzed.

### 4.2. Stress Optimization of Beam-Column Joints of Existing Buildings in Severe Cold Areas

By adopting the static monotonic tensile test method, the moment of force between steel bars and steel plates is increased, and the lap joint model of beam-column joints of existing buildings in cities in severe cold areas is constructed [20]. The index of lap joint position change is expressed as follows:

(8) $$\begin{array}{c} I_{s}=\frac{\mu_{j}A_{j}}{\sum W^{\prime }}F, \end{array}$$

where *I*_*s*_ is the vertical and horizontal spacing, *μ*_*j*_ is the distribution of compressive stress–strain relationship, *A*_*j*_ is stress–strain under uniaxial compression, *W*′ is the parameter value of uniaxial tension descending section, *F* is the biaxial compressive yield strength.

When *F* is 0.1, the biaxial compressive yield strength obtained satisfies:

(9) $$\begin{array}{c} I_{s}=\frac{\lambda_{n}f_{vk}\left(nA_{c}+A_{w}\right)}{\omega \sum A_{f}}, \end{array}$$

where *λ*_*n*_ is the uniaxial tensile strength of beam-column joints of existing buildings in cities in severe cold areas [21, 22], *f*_*vk*_ is the standard value of the parameter value of uniaxial tension descending section, *ω* is the deviation value of flow potential; *A*_*c*_, *A*_*w*_ are the cross-section parameters and distribution area of concrete restrained by stirrups, and ∑*A*_*f*_ is the stiffness recovery coefficient. N is the initial elastic modulus of steel [23, 24].

According to the supporting sequence of the bolt body, the concrete supporting column project is adopted to realize the analysis of the stress structure parameters of the beam-column joints of existing buildings in cities in severe cold areas. In the steel-inserted anchorage joints, the bearing capacity of the specimens is analyzed, and the specific operation process is shown in Figure 3.

To sum up, to realize the equal strength connection of beam-column joints of existing buildings in cities in severe cold areas, the static monotonic tensile test method [25, 26] is adopted to realize the green energy-saving ecological transformation of existing buildings in cities in severe cold areas. The node optimization model is shown in Figure 4.

## 5. Test

In the experimental test of green energy-saving ecological transformation of existing buildings in cities in severe cold areas, the strength grade of steel bars is set to HRB400, and the ultimate strength detection model of beam-column joints of existing buildings in cities in severe cold areas is established by using I-beam, steel tube, and internal reinforcement design method. The yield prestress degree is 234.1 MPa and 232.0 MPa. See Table 1 for the distribution of performance evaluation index system of beam-column joints of existing buildings in severe cold areas.

According to the parameter evaluation index system in Table 1, pin holes with a length of 150 mm, a width of 200 mm and a depth of 150 mm are opened in the brick wall at the top of the horizontal post-pouring belt, with a spacing of 675 mm. The holes are equipped with 4q8 longitudinal reinforcement and 8@100 stirrups, which are poured together with the post-pouring belt, thus connecting the precast reinforced concrete slab with the plain brick wall. Two I-beams are embedded in the bottom of the precast reinforced concrete slab, which are used for positioning the precast wallboard and connected with the substructure. At the top of the precast reinforced concrete slab, a steel bar planting hole is drilled, which is located in the middle of the slab, and an 8-bar is implanted in the hole, with the implantation depth of 80 mmo. The stress analysis of energy-saving ecological transformation is carried out in the green plastic damage model of existing buildings in cities in severe cold areas is shown in Figure 5.

In Figure 5, the stress conditions of the proposed method, reference [9] method and reference [10] method are compared respectively.

According to the stress analysis in Figure 5, the tensile resistance and yield stress of the proposed method are between 0.45∼1.3 kN and 5∼90 kN respectively. The tensile resistance and yield stress of reference [9] method and reference [10] method are between 0.57∼1.23 kN and 12∼78 kN, 0.5∼1.19 kN and 21∼72 kN, respectively. From the above data, it can be seen that the tensile resistance and yield stress expansibility of the proposed method are better. That is, the proposed method can effectively improve the bearing capacity of the reconstructed buildings by establishing the connection model between the concrete foundation of the beam-column joints and the double steel plate composite wall joints of the existing buildings in the severe cold areas, as well as the embedded anchoring and embedded anchoring methods.

The steel bars are planted on the brick wall at the post-cast strip. The depth of the holes for planting steel bars is 200 mm, and the spacing is 300 mm. An 8-screw with an implanted depth of 150 mm is arranged in the hole, which is anchored by pouring steel bar glue, and 180 mm is thrown out of the hole. Eight long-length steel bars are placed in the post-cast strip, and the long-length steel bars are tied together with the bolts implanted in the wall. At the same time, the hooks of the embedded steel bars at the bottom of the precast reinforced concrete slab hook the long-length steel bars. This test is loaded in the vertical and horizontal directions, and a jack is used to apply a constant vertical force of 30 t to the steel beam. The load is transmitted to the concrete loading beam at the top of the test body through the loading steel beam, and then to the specimen to ensure that the axial force is evenly transmitted to the specimen. Load horizontally with electrohydraulic servo actuator and adopt displacement control, and get the comparison of force characteristics of existing buildings in cities in severe cold areas after green energy-saving ecological transformation, as shown in Figure 6.

According to the analysis of Figure 6, in the 10 experiments of the proposed method, after applying a constant vertical force of 30t, the yield stress and tensile resistance always remained above 60, and fluctuated between 60 and 72, with small fluctuations. Therefore, the mechanical reliability of beam-column joint fixation of green building by this method is better. The main reason is that the embedded anchoring method is used in this paper to optimize the shear performance of existing buildings, combined with prestressed reinforcement analysis and yield response analysis.

The yield response of beam-column joints of green buildings is tested. The comparison of cloud pictures of green energy-saving ecological transformation of existing buildings in cities in severe cold areas is shown in Figure 7.

In Figure 7, the more red areas, the higher the heat dissipation capacity of the reconstructed building. That is, the more blue areas, the better the thermal insulation performance of the reconstructed building.

It can be seen from Figure 7 that after the green and energy-saving ecological transformation of existing buildings in cities in severe cold areas by this method, the blue areas have increased significantly. Therefore, this method not only improves the stability of beam-column elements of existing buildings in cities in severe cold areas, but also improves the thermal insulation performance of buildings.

## 6. Conclusions

This paper puts forward the green energy-saving and ecological transformation methods of existing buildings in cities in severe cold areas. The connection model between concrete foundation and double steel plate composite wall of beam-column joints of existing buildings in cities in severe cold areas is established, which improves the bearing capacity of buildings. Combined with embedded anchoring and embedded anchoring methods, the mechanical reliability of beam-column joint fixation is optimized. The embedded anchoring method improves the stability and thermal insulation performance of the building.

Since the weather environment in most cities in China is hot in summer and cold in winter, this study is only aimed at the reconstruction of existing buildings in cities in cold regions. Therefore, the next research will start from the energy-saving transformation of the building envelope, energy-saving transformation of existing buildings in hot summer and cold winter areas.

## Figures and Tables

**Figure 1:** Axis model verification process diagram. (a) Residential area 1. (b) Residential area 2.

**Figure 2:** Relationship between compressive stress and compressive strain.

**Figure 3:** Stress structure parameter analysis process.

**Figure 4:** Distribution optimization of green energy-saving ecological transformation of existing buildings in cities in severe cold areas.

**Figure 5:** Stress analysis of energy-saving ecological transformation. (a) Stretching resistance. (b)Yield stress.

**Figure 6:** Comparison of stress characteristics of existing urban buildings after green energy-saving ecological transformation in severe cold areas.

**Figure 7:** Test on the effect of green energy-saving ecological transformation of existing buildings in cities in severe cold areas. (a) Before transformation. (b) After transformation.

**Table 1:** Performance evaluation index system of beam-column joints of existing buildings in cities in severe cold areas.

Limit strain index layer (weight of comprehensive thermal insulation capacity)	Level 3 indicators (weight of level 2 indicators)
Ultimate strain capacity (042)	Bearing capacity of steel structure (0.345)
	Bearing capacity at the limit point (0.4121)
	Linear arrangement (0.321
	Building regularity (0.126)
	Integral shell structure (0.348)

Building materials (0.26)	Concrete (0.35)
	Constitutive model of prestressed reinforcement (0.123)
	Monotonic loading (0.343)

Proportional stress capacity requirement (0.32)	Peak load (0.55)
	Reverse reload depth (0.234)

## Data Availability

The raw data supporting the conclusions of this article will be made available by the authors, without undue reservation.
